# The Synthesis of Hydroxyapatite by Hydrothermal Process with Calcium Lactate Pentahydrate: The Effect of Reagent Concentrations, pH, Temperature, and Pressure

**DOI:** 10.1155/2022/3481677

**Published:** 2022-03-25

**Authors:** Piotr Szterner, Monika Biernat

**Affiliations:** ŁUKASIEWICZ Research Network, Institute of Ceramics and Building Materials, Ceramic and Concrete Division in Warsaw, Biomaterials Research Group, Postępu 9, Warsaw 02-676, Poland

## Abstract

Hydroxyapatite and other calcium phosphates in the form of whiskers are lately widely considered as fillers for biocomposites due to their special biological and reinforcing properties. Depending on the method of synthesis, apatite whiskers of various sizes and phase composition can be obtained. In our work, hydroxyapatite (HAp) whiskers were successfully prepared in reaction between calcium lactate pentahydrate and orthophosphoric acid. The advantage of the proposed technique is the simple but precise control of the HAp crystal morphology and high product purity which is necessary for biomedical applications. The effect of reagent concentrations, pH, reaction temperature, and pressure on HAp whiskers' morphology and composition was investigated. In the result, we obtained hydroxyapatite of different morphology such as whiskers, hexagonal rods, and nanorods. The products were characterized by SEM, XRD, and FTIR. In this work, the synthesis of HAp whiskers by direct decomposition of calcium lactate pentahydrate chelates under hydrothermal conditions was showed for the first time.

## 1. Introduction

Bioactive calcium phosphate (CaP) ceramics exhibit excellent biocompatibility due to their chemical and crystallographic similarities with the mineral constituents of bones and teeth. The most widely used representative in the CaP group is hydroxyapatite (HAp), (Ca_10_(PO_4_)_6_(OH)_2_) [1]. HAp is the main bone mineral component and typically exhibits excellent bioactivity and osteoconduction [2]. The size and shape of hydroxyapatite particles are closely related to their properties and have an impact on specific applications, especially in the field of biomedicine, as bone fillers in bone tissue engineering, as bioactive coatings, as components of composites, or active substance delivery systems [3–5].

It is known that synthetic hydroxyapatite is often utilized as a biocompatible reinforcement for orthopaedic biomaterials and can provide improved mechanical properties in reinforced polymer composites [6, 7]. The shape, size, and orientation of the filler play a very important role in strengthening composites, and the most effective additives are 2D-shaped fillers, less effective are 1D-shaped fillers, and the least effective are the fillers with the sphere shape [8–10]. Therefore, the synthetic HAp in the form of whiskers could be of particular importance as reinforcing fillers for polymer-ceramic composites, while weaker strengthening properties are demonstrated by hydroxyapatite in the other forms: sphere, rod, and flake [11]. The addition of HAp whiskers to, for example, the dense PAEK composites results in improved tensile and fatigue properties compared to conventional HAp powders, at a given level of reinforcement in polymers, showing mechanical properties similar to those of human cortical bone tissue [12–15].

Nanoscale hydroxyapatite crystals however show better mechanical properties, greater bioactivity, and faster resorption than microcrystals [16]. The sphere-shaped nanoparticles and nanorods can be used for cell targeting and drug and gene delivery [17–19]. Of particular importance are the three-dimensional particles with a mesoporous structure in the form of hollow spheres, in which a high packing of, for example, a drug inside the structure can be obtained. Because of their high specific surface area and porosity, such particles may exhibit favorable and controlled drug release properties [20–22]. Hydroxyapatite can be synthesized using different techniques such as precipitation [23–26], hydrolysis [27, 28], sol-gel method [29, 30], microwave-assisted techniques [31–33], molten salt method [34], hydrothermal synthesis [35–37], and microwave-hydrothermal method [38]or can be extracted from natural resources, e.g., bovine bones, seashells, cockle shells, and egg shells [39–42]. The tendency of HAp to form elongated crystals (whiskers, needles, or rods) was recognized in some of earlier studies on the synthesis of HAp [36, 37].

Hydrothermal synthesis is an important method for obtaining hydroxyapatite in the form of elongated crystals, and it allows the effective control of HAp morphology [43–47]. Hydrothermal process, one of the most common methods for preparation of HAp, is carried out by the reaction of chemicals in aqueous solution at elevated temperature and pressure. Hydrothermal synthesis procedure requires special autoclaves enabling heating of aqueous solutions to high temperatures up to 200°C [16, 48]. Hydrothermal synthesis can also be considered as a chemical precipitation which is conducted at a high temperature, typically above the boiling point of water inside an autoclave or pressure vessel [49]. Depending on hydrothermal reaction conditions, HAp particles with different morphology can be obtained (sphere, microsphere, rod, needle, fiber, whiskers, prism, plate, flake, sheet, bundles of rods or needles or fibers, flower, clusters of nanotubes, oriented bundle, and porous microsphere or mesoporous sphere) [49].

Under the hydrothermal processing, morphology of HAp crystals significantly depends not only on hydrothermal conditions such as processing temperature, reaction time, pH, and additives but also on starting materials [50, 51]. For example, the hydrothermal method of obtaining HAp whiskers from calcium nitrate tetrahydrate, sodium dihydrogen phosphate, and urea as precursors [52] and from calcium hydroxide and calcium hydrogen phosphate dihydrate [51] is known from the literature. The aim of our work was to receive HAp directly from calcium chelate like calcium lactate pentahydrate and orthophosphoric acid and investigate the effects of factors such as reagent concentrations, starting solution pH, reaction temperature, and pressure on HAp morphology and phase composition. The products reported in this part of manuscript were analyzed by means of the following techniques: scanning electron microscope (SEM), X-ray diffraction method (XRD), and Fourier transform infrared spectroscopy (FTIR).

According to literature review, no data about the hydrothermal synthesis with the direct use of calcium lactate pentahydrate have been published. To our knowledge, in this work, for the first time, the effect of reaction condition on whiskers' morphology and their phase composition during decomposition of calcium lactate pentahydrate chelates was showed.

## 2. Experimental

### 2.1. Materials

The main substrates for the synthesis were calcium lactate pentahydrate (C_6_H_10_CaO_6_·5H_2_O) (pure p.a., CAS: 5743-47-5) and orthophosphoric acid (H_3_PO_4_) (pure p.a., CAS: 7664-38-2) from Chempur^®^ Chemical Company, Poland.

### 2.2. Synthesis

The whiskers of HAp were prepared by the hydrothermal method. Synthesis was carried out under various conditions using a stainless steel reactor (Büchiglasuster^®^, miniclave steel type 3/300 ml, 100 bar) enabling heating of aqueous solutions to high temperatures up to 200°C.

HAp whiskers were synthesized from aqueous solutions containing calcium lactate pentahydrate and orthophosphoric acid. The molar ratio of Ca to P in the solution was 1.67, which is equivalent to that of stoichiometric HAp. For all syntheses, the concentration of Ca was in the range from 0.025 to 0.2 mol L^−1^. The calcium lactate pentahydrate was dissolved in deionized water to a homogeneous solution, and then a solution of orthophosphoric acid was added. The mixed solutions were poured into a reaction vessel and heated to the set value of temperature. During hydrothermal synthesis, the temperature and pressure inside of reactor were continuously monitored. Reaction conditions were controlled by using a heating assembly (800 W, Termtech) and temperature controller (RE72, LUMEL). All parameters of heating process (e.g., temperature and heating time) were controlled by Program Lumel Process 1.2 (Lumel S.A. Company, Poland). The reaction temperature was measured by using a thermocouple (TP-234k-b-200; Czaki^®^ Thermo-Product) placed inside a thermowell in the reaction vessel. The pressure inside of reactor was controlled by using the installed manometer.

The reactor with the heating assembly was placed on the magnetic stirrer (IKA^®^, RH basic) with the heating temperature range between 50 and 320°C and speed range from 100 to 2000 rpm. The pH of the starting solutions and solutions after the synthesis was measured with a glass pH electrode (Eutech Instruments, CyberScan PCD 6500) at 25°C. Upon completion of each reaction, the vessel was cooled to ambient temperature (∼25°C) overnight. The product was then filtered off, washed quickly with deionized water four times, and finally dried in air in the laboratory dryer (KCW-100, PREMED) at 100°C for at least 6 h.

### 2.3. Characterization

#### 2.3.1. SEM Analysis

Microscopic observations, sample morphology and local microstructure analysis of the obtained whiskers were performed using a field emission scanning electron microscope (Nova NanoSEM200, FEI). Imaging of sample microstructure was performed in high vacuum conditions using ETD (Everhart-Thornley detector) detector at 10 kV accelerating voltage. Before the study, the samples were covered with conductive material (25 nm gold film) using a sputter coater, Leica EM SCD500. Width and length of the obtained whiskers were determined on the basis of microscopic images using measurement and annotation functions on the sample area.

#### 2.3.2. XRD Measurements

The phase composition of products obtained by hydrothermal synthesis was analysed by the Bragg–Brentano X-ray diffraction method (XRD) on a Bruker-AXS D8 DAVINCI diffractometer designed for a copper anode tube. The diffractograms were recorded in an angular range from 10° to 80° 2*θ* (Cu K*α*), measuring Step 0.01 and measurement time: 1 s/step. The diffractometer's optical system was composed of a 0.3-inch divergence slot, a 1.50 antiscatter slot, two 2.5 Soller slots, a Ni filter, and a LYNXEYE strip detector with 2.94 field of view. Crystalline phases were identified in DIFFRACplus EVA-SEARCH software with recorded diffraction patterns and standards from ICDD PDF-2 and PDF-4+ 2016 databases and the Crystallography Open Database (COD). Quantitative analysis was carried out using the Rietveld method in the TOPAS v.50 software, based on published crystalline structures (COD).

Before X-ray analysis, all HAp samples were easily ground manually by using a mortar and pestle. In the case of small amounts of some samples, the preparations were prepared by obtaining an alcohol-based suspension with the tested powder, pouring the suspension onto a nonreflective table and evaporating the solvent.

#### 2.3.3. FTIR Analysis

Functional groups of the samples were identified by Fourier transform infrared spectroscopy (FTIR). Measurements of absorbance were made using a TENSOR 27 (Bruker) equipped with a DLaTGS detector. The analysis was performed in the wavelength range from 400 cm^−1^ to 4000 cm^−1^. The samples were prepared as pressed pellet-shaped KBr moulds.

## 3. Results

### 3.1. Synthesis

The synthesis was carried out under various conditions. During the synthesis, the following experimental parameters were changed independently: time of the synthesis (3 h, 5 h, and 7 h), temperature (130°C, 150°C, 170°C, and 200°C), and pH of the reaction solution (3.91–11.06). The Ca^2+^ ion concentrations in starting synthesis solutions were changed in the range between 0.025 mol/dm^3^ and 0.2 mol/dm^3^. The molar Ca/P ratio in starting solutions was 1.67, which is equivalent to that of stoichiometric HAp. The effect of selected parameters on the morphology and phase composition of the obtained products is presented in Table 1.

### 3.2. The Effect of Ca^2+^ Ions Concentration and pH of Starting Synthesis Solution on the Obtained Products' Character

The effect of Ca^2+^ ions concentration on the morphology and phase composition of products was determined for synthesis carried out at a temperature of 200°C, under a pressure of 20 bar, and at a pH about 4. The Ca^2+^ concentration in starting reaction solution was 0.025 mol/dm^3^, 0.05 mol/dm^3^, 0.1 mol/dm^3^, and 0.2 mol/dm^3^, respectively. For comparison, reactions with each of the abovementioned Ca^2+^ concentration were carried out at two different times: 3 h and 5 h. Moreover, for two selected Ca^2+^ concentrations (0.05 mol/dm^3^ and 0.1 mol/dm^3^), the synthesis was carried out in time of 7 hours. The various conditions, phase composition, morphology, length, and width of the obtained products are given in Table 1 (I).

The product of all mentioned reactions was pure HAp. Sample diffraction patterns of products prepared during 5 h from starting synthesis solutions with Ca^2+^ concentrations in the range of 0.025–0.2 mol/dm^3^ are shown in Figure 1.

All signals on the presented diffraction patterns are in good agreement with characteristic signals from pure hydroxyapatite in reference model (PDF no. 00-09-0432). No signals from impurities were observed. Despite that the Ca^2+^ concentrations used in the synthesis did not affect the phase composition, the morphology of the obtained products varied with the various Ca^2+^ concentrations. The obtained HAp particles were formed in two crystal structures similar to whiskers or hexagonal rods. The SEM images of products obtained during 5 hours of synthesis are presented in Figure 2. The products in the form of whiskers were obtained for Ca^2+^ concentrations of 0.025 mol/dm^3^ and 0.05 mol/dm^3^ (Figures 2(a) and 2(b)). Moreover, the product for synthesis with a Ca^2+^ concentration of 0.05 mol/dm^3^ occurs in whisker form, created characteristic sheaf bundles (Figure 2(b)). For synthesis with a Ca^2+^ concentration of more than 0.1 mol/dm^3^ (Figures 2(c) and 2(d)), the product in the form of hexagonal rods was obtained.

Ca^2+^ concentration of starting synthesis solution also affected the particles' dimensions. The mean length of the whiskers prepared in a time of 5 hours from the solution with Ca^2+^ concentrations of 0.025 mol/dm^3^ and 0.05 mol/dm^3^ (40–111 *μ*m) was higher than the length of hexagonal rods prepared from the solution with a Ca^2+^ concentration of 0.1–0.2 mol/dm^3^ (15–38 *μ*m).

Similar relationships were observed for the synthesis carried out during 3 hours. As can be seen in Figure 3(a), the whiskers were obtained only for the synthesis with the Ca^2+^ concentration of 0.025 mol/dm^3^. The mean length of the whiskers was in the range of 63.5–96.2 *μ*m. They were longer than hexagonal rods obtained in the case of synthesis with the Ca^2+^ concentration of 0.05 – 0.2 mol/dm^3^ (10–30 *μ*m) (Figures 3(b)–3(d)). It was observed for 3 hours of synthesis that, with the increase of Ca^2+^ concentration in starting solution, the hexagonal rods' length increased slightly. However, the last relationship was not observed for the 5-hour synthesis as well as the 7-hour synthesis (Table 1 (I)).

In addition, for the Ca^2+^ concentration of 0.05 mol/dm^3^ and with a synthesis time of 5 h and a temperature of 200°C, the relationship of phase composition and shape of the obtained products to the pH of the starting reaction solution was examined (Table 1 (II)). The XRD patterns of the reaction products obtained from starting solutions with pH values of 3.9, 9.3, and 11.1 are shown in Figure 4. For each of the pH values, the diffraction patterns of the reaction products show only the characteristic signals from pure hydroxyapatite in accordance with the standard (PDF no. 00-09-0432). No signals from any impurities were present. As can be seen in Table 1 (II) and Figure 2(b), HAp in the form of whiskers was formed only in the case of a reaction carried out at pH = 3.9. In other cases, the products in the form of aggregates of various sizes were obtained (Figures 2(e) and 2(f)).

FTIR analyses of samples obtained in 5-hour hydrothermal synthesis carried out at 200°C and pH about 4, from starting solutions with the Ca^2+^ concentration of 0.05, 0.1, and 0.2 mol/dm^3^, and FTIR spectrum of sample obtained under identical conditions but in pH = 11.06 are shown in Figure 5. The spectra show characteristic bands corresponding with functional groups of hydroxyapatite [38, 53–55].

The absorption bands at 3571 and 634 cm^−1^ are assigned to stretching mode (*ν*s) and vibrational mode (*ν*L) of the hydroxyl group (OH) [53, 54]. Bands at 1094, 1046, 1029, 962, 602, 562, and 473 cm^−1^ are assigned to vibrations of the phosphate group (PO_4_). The first peak at 1094 cm^−1^ emanates from a triply degenerated asymmetric stretching mode vibration (*v*_3_) of the P-O bond of the phosphate group. The other two components of this triply degenerated vibration (*v*_3_) of the P-O bond of the phosphate group appear at 1046 and 1029 cm^−1^. The peak at 962 cm^−1^ is assigned to a nondegenerated symmetric stretching mode (*v*_1_) of the P-O bonds of the phosphate group (PO_4_).

The peaks at 602 and 562 cm^−1^ are assigned to a triply degenerated bending mode (*v*_4_) of the O-P-O bonds of the phosphate group. The weak peaks at 473 cm^−1^ are components of the doubly degenerated bending mode (*v*_2_) of the O-P-O bonds of the phosphate group (PO_4_). The peaks at 2000 and 1991 cm^−1^ are assigned to a 2*v*_3_ harmonic overtone or to a combination band (*v*_1_ + *v*_3_). The peaks at 2070 cm^−1^ have been interpreted as combination bands or harmonic overtones. The transmission band at 1647 cm^−1^ was attributed to the H-O-H bending mode of water, indicating the existence of water in the sample [38]. The broad absorption peak at 3400 cm^−1^ is assigned to adsorbed water molecules [54]. The peaks related to gaseous CO_2_ (dissolved) are visible at 2360 and 2341 cm^−1^ [56]. The CO_3_^2−^ group can be incorporated into the structure of HAp and can be located in the position OH (A-type) or PO_4_ (B-type) [57].

In the FTIR spectrum for obtained HAp, lacks of bands at 1420, 1450, and 1545 cm^−1^ characteristic for carbonated hydroxyapatite A-type and lacks of bands at 1420 and 1460 cm^−1^ characteristic for carbonated hydroxyapatite B-type attributed to the CO_3_^2-^ group [55]. Some CO_3_^2-^ derived bands are observed at 874 cm^−1^ [53]. It might be due to the adsorption of atmospheric carbon dioxide during the sample preparation. This small amount of CO_3_^2-^ has not produced either carbonated HAp (as evident by XRD) or other carbonates. This peak also can be assigned to monohydrogen phosphate (HPO_4_^2-^). Also, we can accept that the obtained HAp samples were free of HPO_4_^2-^, as concluded from the infrared spectroscopic data analysis. On the spectra, there is the absence of characteristic detectable peaks for HAp in the presence of dihydroxy phosphates in the crystal lattice at wavelengths of 868, 1215, or 2400 cm^−1^ [54].

In several FTIR spectra, particularly for hydroxyapatite obtained at pH 11.06 (Figure 4), the presence of organic material (C-H) is detected as low intensity peaks at range 2840–3000 cm^−1^. There are peaks which are characteristic of stretching vibrations from C-H bonds [58, 59]. According to this FTIR study, it can be indicated that a small amount of derivative of lactate adheres to the surface of the final product. Based on those results, it can be stated that, in the hydrothermal synthesis from calcium lactate pentahydrate and orthophosphoric acid, the pure hydroxyapatite was obtained.

### 3.3. The Effect of Temperature and Pressure on the Obtained Products' Character

In order to determine the effect of temperature and pressure of reaction on the kind of product, synthesis was carried out in one time of 5 h, in pH about 4, with the same fixed Ca^2+^ concentration of 0.05 mol/dm^3^, at different temperatures of 200°C, 170°C, 150°C, and 130°C, and corresponding pressures of 20 bar, 10 bar, 6 bar, and 4 bar, respectively. The results of synthesis are presented in Table 1 (III). SEM images of the obtained products are presented in Figure 6. XRD patterns confirming the phase compositions of the obtained products are shown in Figure 7.

For synthesis at temperatures of 200°C, 170°C, and 150°C, all diffraction peaks can be indexed and assigned to a pure HAp phase. The results of this analysis are consistent with the reference data (PDF no. 00-009-0432). Moreover, the diffraction pattern of product obtained at 130°C can be assigned to a pure monetite (CaHPO_4_), which is in good agreement with the reference data (Cod no. 9007619) [60].

As can be seen, the reaction temperature had obvious effects on the phase composition, form, and dimensions of products. For the lowest of tested temperatures and pressures (130°C and 4 bar), calcium hydrogen phosphate (monetite) in characteristic plate form was obtained as a product. For reactions carried out at 150°C and higher, pure HAp in whisker form was obtained. As the temperature and pressure of the reaction increased, the length of the obtained whiskers also increased (Figure 6). In the case of the synthesis carried out at 200°C and in pressure of 20 bar, HAp whiskers reached the length in a range of 58.4–111.1 *µ*m.

FTIR analyses of two samples obtained from the solution with the Ca^2+^ concentration of 0.05 mol/dm^3^ in a time of 5 h and at temperatures of 200°C and 130°C are presented in Figure 8. The FTIR study conﬁrmed the presence of hydroxyapatite and monetite that was identiﬁed by XRD. The FTIR spectrum shows characteristic bands of corresponding functional groups relative to hydroxyapatite [53–55] and monetite [61–64].

The spectrum obtained for HAp (Figure 8(a)) is typical for stoichiometric HAp, as described above. In the monetite spectrum (Figure 8(b)), three different types of H-bonds, characteristic of this mineral, were observed [61]. The H-bonds may be related to stretching (P)O-H vibration bands at approximately 2360, 2850, and 3200 cm^−1^. Moreover, other broad bands can be observed. The broad band at approximately 3440 cm^−1^ is related to O-H stretching of residual-free water. The broad band between 1600 and 1700 cm^−1^ is related to H-O-H bending and rotation of residual-free water. The broad band located between 1300 and 1450 cm^−1^ is associated to P-O-H in plane bending. Regarding the phosphate functional group, intense bands at 1130, 1066, and 995 cm^−1^ related to the P-O stretching (*v*_3_, *v*_3_, *v*_1_) and the band at 889 cm^−1^ related to the P-O(H) stretching (*v*_3_) were observed. The bands at 563 and 534 cm^−1^ are due to O-P-O(H) bending mode (*v*_4_, *v*_4_), while the 432 cm^−1^ band is due to the O-P-O bending mode (*v*_2_). Similar to spectrum FTIR obtained for hydroxyapatite, the peaks at 2360 and 2341 cm^−1^ can be related to gaseous CO_2_ (dissolved) [56].

## 4. Discussion

### 4.1. Synthesis

General reaction during the hydrothermal synthesis of hydroxyapatite from calcium lactate pentahydrate and orthophosphoric acid is presented below (reaction (1)). The synthesis is based on thermal decomposition of calcium chelates under specific conditions (high temperature and high pressure). In the first step of the process, calcium ions (Ca^2+^) are formed (reaction (2)), which next react with the phosphate groups (PO_4_^−3^) and hydroxyl groups (OH^−^) (reaction (3)) [36, 65].

(1) $$\begin{array}{c} 10{\left[{\text{CH}}_{3}\text{CH}\left(\text{OH}\right)\text{COO}\right]}_{2}\text{Ca}\cdot 5{\text{H}}_{2}\text{O}+6{\text{H}}_{3}{\text{PO}}_{4}⟶20{\text{ CH}}_{3}\text{CH}\left(\text{OH}\right)\text{COOH}+{\text{Ca}}_{10}{\left({\text{PO}}_{4}\right)}_{6}{\left(\text{OH}\right)}_{2}+48{\text{H}}_{2}\text{O}, \end{array}$$

(2) $$\begin{array}{c} {\left[{\text{CH}}_{3}\text{CH}\left(\text{OH}\right)\text{COO}\right]}_{2}\text{Ca}\cdot 5{\text{H}}_{2}\text{O}⟶{\text{Ca}}^{2+}+\;2{\text{CH}}_{3}\text{CH}\left(\text{OH}\right){\text{COO}}^{-}+5{\text{H}}^{+}+5{\text{OH}}^{-}, \end{array}$$

(3) $$\begin{array}{c} 10{\text{Ca}}^{2+}+6{\text{PO}}_{4}^{3-}+2{\text{OH}}^{-}⟶{\text{Ca}}_{10}{\left({\text{PO}}_{4}\right)}_{6}{\left(\text{OH}\right)}_{2}. \end{array}$$

Depending on the concentration of Ca^2+^ ions in the starting solution, on the temperature of the process, and on its time, products with different phase composition and different morphology can be obtained (Table 1) [36].

### 4.2. The Effect of Process Conditions on Properties of the Obtained Products

According to Table 1 (I) and Figure 1, Ca^2+^ concentrations used in the synthesis did not affect the phase composition. All signals on the diffraction patterns are in good agreement with characteristic signals from pure hydroxyapatite in the reference model (PDF no. 00-09-0432). The most visible signals for hydroxyapatite are the characteristic signals for 2*θ* degree equal to 31.80 and 32.90 corresponding to crystallization planes (211) and (300), respectively. According to literature data, the (300) peak becomes the strongest when HAp whiskers grow along the *c*-axis [66, 67]. However, in Figure 1, differences between diffraction peaks (211) and (300) are visible. For the Ca^2+^ concentrations of 0.025 and 0.1 mol/dm^3^, the strongest diffraction peak is (300) and the second strongest peak is (211), but for the Ca^2+^ concentrations of 0.05 and 0.2 mol/dm^3^, the strongest diffraction peak is (211) and the second strongest peak is (300). The morphology of the obtained products varied with the various Ca^2+^ concentrations (Figure 2) [66, 67].

Ca^2+^ concentration of starting synthesis solution also affected the particles' dimensions. From the results obtained, it is particularly clear that HAp particles obtained in form of whiskers are much longer than HAp obtained in form of hexagonal rods. According to the literature [36], decreasing the concentration of Ca^2+^ resulted in a slower release of calcium ions from solution and a decreased nucleation rate of crystals which were able to grow to a greater length and form whiskers.

In our research, for the hydrothermal reaction between calcium lactate pentahydrate and orthophosphoric acid, the influence of temperature and pressure on the morphology and phase composition of the products is also noticeable. The pure hydroxyapatite phase was obtained for the temperature of 150°C and higher, and HAp whiskers were obtained at a temperature of 200°C and a pressure of 20 bar. These data are in accordance with other literature reports. Kimn and Ohtsuki [50] showed that, in the case of hydroxyapatite formation from calcium carbonate, the size of the needle crystals that were formed during the process increased with increasing temperature. On reaching a temperature of 200°C, plate-shaped HAp was observed [50].

As can be seen also in Figure 2, the change in pH of the reaction solution affected the shape of the obtained HAp particles. These observations are consistent with the studies by Liu et al., who also showed that, in hydrothermal synthesis of hydroxyapatite using Ca(OH)_2_ and CaHPO_4_·2H_2_O, the pH value is a significant parameter variable in altering the hydroxyapatite morphology [51]. In our research, for more basic medium (pH = 9.3 and 11), quite different products in the form of aggregates consisting of nanorods of hydroxyapatite can be obtained. By appropriately changing the pH and the concentration of Ca^2+^ ions, hydroxyapatite particles of the selected shape (whiskers, hexagonal rods, and nanorods) can be obtained in the presented hydrothermal method, even while maintaining the same temperature, pressure, and reaction time (Figure 9).

However, pH of the reaction solution did not affect the phase composition of the reaction products (Figure 4). In Figure 4, it can further be seen that, for pH = 3.9, sharp peaks appeared mainly. This can suggest that the obtained sample was well crystallized. However, the HAp powders obtained from the solution with pH = 9.1 and pH = 11.1 showed comparatively lower and less sharp signals. While maintaining the same amounts of material tested and the same conditions for XRD analysis, this may suggest lower crystallinity of the products obtained in an alkaline environment. Hence, it can be assumed that the differences in crystallinity observed on the XRD patterns (Figure 4) confirm the different forms of the obtained HAp particles (Figure 2). From the results obtained and the data contained in Table 1, it can be concluded that the results obtained are affected by many factors at the same time. For example, the dimensions of the obtained particles cannot be compared solely for the sole change in Ca^2+^ concentration. The form of particles formed in the *in situ* reaction plays a big role. Some concentrations are insufficient to obtain well-formed particles, for which an analysis of the dependence on a given factor can be performed.

## 5. Conclusions

In this work, fibrous hydroxyapatite was successfully prepared in reaction between calcium lactate pentahydrate and orthophosphoric acid. The advantage of the proposed technique is the simple but precise control of the HAp crystal morphology. The effect of reagent concentrations, pH, reaction temperature, and pressure on HAp whiskers' morphology and composition was investigated.

The presented results show influence of concentration of calcium (Ca^2+^) on the morphology of the obtained product. The products in the form of whiskers of hydroxyapatite were obtained during hydrothermal synthesis for concentrations of calcium Ca^2+^ = 0.025 mol/dm^3^ and Ca^2+^ = 0.05 mol/dm^3^, at a final temperature of 200°C under pressure 20°bar, which was held for 5 hours, with the stirring rate of 250 rpm and with the reaction heating rate of 2.5°C/min. For concentrations of calcium Ca^2+^ = 0.1 mol/dm^3^ and Ca^2+^ = 0.2 mol/dm^3^, the product was obtained in the form of hexagonal rods.

Length of the whiskers increase with decrease in the concentration of calcium. The mean length of whiskers prepared in the concentrations of Ca^2+^ = 0.025 mol/dm^3^ and Ca^2+^ = 0.05 mol/dm^3^ in the time of 5 hours was in the range of 40–111 *μ*m, and it was bigger than the length of hexagonal rods prepared in the concentration of Ca^2+^ = 0.1–02 mol/dm^3^ (15–38 *μ*m). The products in the form of whiskers were obtained for 3 hours of synthesis and the concentration of Ca^2+^ = 0.025 mol/dm^3^. For concentrations of Ca^2+^ = 0.05–0.2 mol/dm^3^, the product was obtained in the form of hexagonal rods, not exactly formed, which suggests that the time of 3 hours is not enough for complete growth. Noticeable in the hydrothermal reaction between calcium lactate pentahydrate and orthophosphoric acid was also influence of temperature and pressure on the morphology and phase composition of the products.

The product in the form of pure HAp whiskers was observed at a temperature of 200°C and a pressure of 20 bar. At the temperature of 170°C and 150°C and the pressure of 10 and 6 bar, hydroxyapatite in the form of hexagonal rods was obtained. The pure calcium hydrogen phosphate (monetite) was formed during the synthesis at the temperature of 130°C and the pressure of 4 bar, which suggests that the temperature for synthesis of HAp should be more than 130°C. The advantage of this presented method is obtaining pure hydroxyapatite of different morphology without the use of organic additives that can contaminate the product. In this work, the synthesis of HAp whiskers by direct decomposition of calcium lactate pentahydrate chelates under hydrothermal conditions was showed for the first time.

The presented method enables obtained hydroxyapatite of different morphology such as whiskers, hexagonal rods, and nano rods, which can be used like fillers in composites applied in biomaterials.

## Figures and Tables

**Figure 1:** The XRD patterns of HAp obtained during 5 h reaction, at 200°C, from starting synthesis solutions with different Ca^2+^ concentrations.

**Figure 2:** SEM images of products obtained in hydrothermal synthesis (200°C, 20°bar, 5°h) for (a) Ca^2+^ concentration 0.025 mol/dm^3^ and pH 4.20, (b) Ca^2+^ concentration 0.05 mol/dm^3^ and pH 3.91, (c) Ca^2+^ concentration 0.1 mol/dm^3^ and pH 4.13, (d) Ca^2+^ concentration 0.2 mol/dm^3^ and pH 4.20, (e) Ca^2+^ concentration 0.05 mol/dm^3^ and pH 9.3, and (f) Ca^2+^ concentration 0.05 mol/dm^3^ and pH 11.06 (magnification of 2500×).

**Figure 3:** SEM images of products obtained in hydrothermal synthesis (200°C, 20 bar, 3°h) for (a) Ca^2+^ concentration 0.025 mol/dm^3^ and pH 3.77, (b) Ca^2+^ concentration 0.05 mol/dm^3^ and pH 4.08, (c) Ca^2+^ concentration 0.1 mol/dm^3^ and pH 3.69, and (d) Ca^2+^ concentration 0.2 mol/dm^3^ and pH 3.99 (magnification of 2500×).

**Figure 4:** XRD patterns of HAp powders synthesized during 5 h at a temperature of 200°C from starting solutions with the Ca^2+^ concentration of 0.05 mol/dm^3^ with different pH values.

**Figure 5:** FTIR spectra of hydroxyapatite obtained in 5-hour hydrothermal synthesis at a temperature of 200°C and pH about 4, from the solution with the Ca^2+^ concentration of (a) 0.05 mol/dm^3^, (b) 0.1 mol/dm^3^, and (c) 0.2 mol/dm^3^, and in 5-hour hydrothermal synthesis at a temperature of 200°C and pH = 11.06, from the solution with the Ca^2+^ concentration of (d) 0.05 mol/dm^3^.

**Figure 6:** SEM images of products obtained in hydrothermal synthesis (Ca^2+^ concentration of 0.05 mol/dm^3^, 5 h, pH about 4) for (a) 200°C and 20 bar, (b) 170°C and 10 bar, (c) 150°C and 6 bar, and (d) 130°C and 4 bar (magnification of 2500×).

**Figure 7:** XRD patterns of products obtained in hydrothermal synthesis carried out at different temperatures (Ca^2+^ concentration of 0.05 mol/dm^3^, 5 h, pH about 4).

**Figure 8:** FTIR spectra of hydroxyapatite (a) and monetite (b) obtained at temperatures of 200°C and 130°C, respectively, in 5-hour hydrothermal synthesis from the solution with the Ca^2+^ concentration of 0.05 mol/dm^3^.

**Figure 9:** SEM images of products obtained in hydrothermal synthesis (200°C, 20°bar, 5°h) for (a) whiskers (Ca^2+^ concentration 0.05 mol/dm^3^ and pH 3.1), (b) hexagonal rods (Ca^2+^ concentration 0.2 mol/dm^3^ and pH 4.20), and (c) nanorods (Ca2+ concentration 0.05 mol/dm3 and pH 9.0) ((a) and (b), magnification of 1000×; (c), magnification of 100000×).

**Table 1:** The effect of hydrothermal synthesis conditions on the morphology and phase composition of the obtained products.

Ca^2+^ concentration (mol L^−1^)	pH before synthesis	Time of synthesis (h)	Temperature of synthesis (C)	Pressure (bar)	Stirring rate (rpm)	The reaction heating rate (C/min)	The obtained whiskers' length (*µ*m)	The obtained whiskers' width (*μ*m)	Phase composition (form)
*(I) Different Ca* ^*2+*^ *concentrations*									
0.025	3.77	3	200	20	250	2.5	63.5–96.2	2.0–5.4	HAp (whiskers)
0.05	4.08	3	200	20	250	2.5	10.0–22.0	2.0–3.0	HAp (hexagonal rods)
0.1	3.69	3	200	20	250	2.5	13.6–25.0	1.8–5.0	HAp (hexagonal rods)
0.2	3.99	3	200	20	250	2.5	18.2–30.0	2.3–4.5	HAp (hexagonal rods)
0.025	4.20	5	200	20	250	2.5	40.6–82.9	2.0–4.3	HAp (whiskers)
0.05	3.91	5	200	20	250	2.5	58.4–111.1	2.0–3.0	HAp (whiskers)
0.1	4.13	5	200	20	250	2.5	30.2–37.8	2.2–4.5	HAp (hexagonal rods)
0.2	4.20	5	200	20	250	2.5	15.5–20.0	2.3–3.4	HAp (hexagonal rods)
0.05	4.08	7	200	20	250	2.5	27.8–69.5	1.5–5.5	HAp (hexagonal rods)
0.1	3.94	7	200	20	250	2.5	21.1–56.8	2.2–5.5	HAp (hexagonal rods)

*(II) Different pH of reaction solution*									
0.05	3.91	5	200	20	250	2.5	58.4–111.1	2.0–3.0	HAp (whiskers)
0.05	9.3	5	200	20	250	2.5	Aggregates of various sizes, nanorods length 114.9–230 nm, width 41.2–92.0 nm		HAp (aggregates consisting of nanorods)
0.05	11.06	5	200	20	250	2.5	Aggregates of various sizes		HAp (aggregates consisting of nanorods)

*(III) Different temperature and pressure of synthesis*									
0.05	3.91	5	200	20	250	2.5	58.4–111.1	2.0–3.0	HAp (whiskers)
0.05	3.77	5	170	10	250	2.5	39.0–66.8	1.5–4.9	HAp (hexagonal rods)
0.05	3.83	5	150	6	250	2.5	27.8–65.4	2.2–6.6	HAp (hexagonal rods)
0.05	3.95	5	130	4	250	2.5	22.2–44.4	27.8–38.9	Monetite (plate formations)

## Data Availability

The data generated during this study are available at ŁUKASIEWICZ Research Network, Institute of Ceramics and Building Materials, Ceramic and Concrete Division in Warsaw, Biomaterials Research Group, Postępu 9, Warsaw, 02-676, Poland, and are available from the corresponding author upon request.
